RETRACTED

# Internet-based supply chain financing-oriented risk assessment using BP neural network and SVM

**DOI:** 10.1371/journal.pone.0262222

**Published:** 2022-01-21

**Authors:** Weiqiong Fu, Hanxiao Zhang, Fu Huang

**Affiliations:** 1 School of Economics and Management, Huizhou University, Huizhou, China; 2 School of Accounting, Guangzhou Huashang College, Guangzhou, China; Ministry of Natural Resources North Sea Bureau, CHINA

## Abstract

To better prevent the potential risks in Internet-based Supply Chain Financing (SCF) products, this paper optimizes and evaluates the Internet-based SCF-oriented Credit Risk Evaluation (CRE) method. Firstly, this paper summarizes 12 risk factors of SCF business, establishes a Risk Assessment Index System (RAIS) with good consistency and stability; then, the principles of Backpropagation (BP) Neural Network (NN) is expounded together with Support Vector Machines (SVM) and Genetic Algorithm (GA) model. Consequently, a CRE model is implemented by the NN tools in MATLAB based on the collection of multiple groups of SCF-oriented risk assessment samples. Subsequently, the assessment samples are trained and tested. Finally, the SCF-oriented CRE model is proposed and verified. The results show that the BP-GA model has presented high prediction consistency with the actual classification. According to the comparison of classification results of SVM, BP model, and BP-GA model, the classification accuracy of test samples of the proposed Internet-based SCF-oriented CRE system using BP-GA model reaches 97.19%; the Type I and Type II error rate of the CRE system based on BP-GA model is 7.2% and 14.21%, respectively. Therefore, a suitable SCF-oriented CRE method is put forward for China’s commercial banks along with scientific and feasible suggestions to manage SCF-oriented credit risks more reasonably and effectively.

## Introduction

Small and Medium-sized Enterprises (SMEs) account for the most in Chinese businesses and, thus, play an absolutely important role in the development of China’s market economy by contributing over 50% of China’s GDP and tax revenue and helping to solve the largest labor employment. SMEs have gradually become the source of vitality of China’s economic development [1, 2]. Yet, some problems have become inevitable. Compared with developed countries, the Sino-firms have a relatively late start, small scale production, and low technical content; meanwhile, their fixed assets are extremely limited and less mortgageable, lack transparent operation or management mechanism, and they often employ chaotic financial systems. Generally, banks promise enterprise loans only on realizable-asset collateral or powerful third-party guarantee. Yet, under such conditions, most Chinese SMEs will be shut out from the financial support of financial institutions, thus limiting their development [3, 4]. For a long time, financing difficulties have always been the obstacles on the path of Chinese SMEs’ advancement; the emergence of Supply Chain (SC) Financing [SCF] might just be tailor-made for this problem. Different from the traditional financial model, the focus of SCF shifts from the financial and asset status of SMEs to the trade authenticity and credit status of SC enterprises to improve the financing efficiency of enterprises and reduce the financing risks [5].

RETRACTED

In terms of the Internet-based SCF risk assessment, Zhang et al. (2021) [6] pointed out that with the implementation of the "Internet +" development strategy, Internet-based SCF technology was gradually becoming the dominant financing approach for SMEs; the close combination of SCF with physical industry and finance had greatly promoted the Sustainable Development (SD) of SC subjects, especially, SMEs. Therefore, by integrating the components and characteristics of BlockChain (BC) into all application links of SCF, the financing difficulties of SMEs in SCF could be effectively solved. Wang et al. (2019) [7] put forward the business processes of three basic financing modes of SCF and the shortcomings in the operation of each mode; then, the risk sources and influencing factors of SCF were analyzed, focusing on the operation risks; finally, combined with the special functions of Internet of Things (IoT) technology and the business process of Inventory Pledge Financing (IPF) mode, a new IPF mode was designed. Yang et al. (2019) [8] proposed an Internet-based SCF risk management model based on data science. Zhang et al. (2021) [9] established the improved Random Forest (RF)-based online SCF-oriented Risk Assessment Index System (RAIS); the data analysis proved the feasibility and accuracy of the proposed system and provided a new method for the SC risk assessment. Sreedharan et al. (2019) [10] argued that SC risks were the major obstacles in operational excellence of organizations; the purpose was to evaluate the SC risk of pharmaceutical industry and its impact on SC operational performance; based on literature review, 44 projects were divided into five aspects: supplier risk, production risk, demand risk, infrastructure risk, and macro risk, based on which a structured Questionnaire Survey (QS) was designed and was distributed over the Internet on the pharmaceutical industry, and the response rate was 66.20%; afterward, the corresponding assumptions between these structures and production risk were tested using structural equation model; the results of structural equation model suggested that except demand risk, all other threats were negatively correlated with production risk; additionally, the organizations were ranked according to their production risk by proposing a SC risk assessment index, which was based on the rating obtained by experts using fuzzy technology. Literature review corroborates that the domestic SCF research is mainly from the perspective of banks, only provide financing services for SMEs. Internationally, the SCF research has a multi-perspective. Overall, the current research on SCF focuses on the conceptual description and operational modes without many systematic and in-depth studies, and some existing problems are prominent. Firstly, there is a lack of empirical research on the implementation effect of SCF; it has been universally believed that SCF can accelerate the working capital turnover of SMEs in the SC and reduce the financing cost, but the research is still in the theoretical discussion stage. There is a lack of in-depth analysis on the impact and degree of the implementation of SCF on SMEs in SC. Secondly, the literature on SCF risk is relatively few, which only gives a general description and does not conduct quantitative research on specific risks; hence, the analysis, identification, evaluation, and control of SCF risks still need to be further studied. Thirdly, in terms of the theoretical research of SCF, the current research on the game relationship between commercial banks, SC-affiliated SMEs, and SC-dominating enterprises is still relatively scarce, and the analysis of the behavior selection mode of various actors in the process of SCF is lacking. Fourthly, China’s research on SCF ignores the role of advanced e-commerce and technical service platform. Only with the help of these platforms can the information flow and capital flow be combined in the SC. The above four aspects need urgent solutions. The further study of SCF is of great significance to the development of SC Management (SCM) theory.

RETRACTED

Therefore, this paper makes an in-depth study on the operation mode of SCF, summarizes the risk factors of multiple SCF businesses, establishes the RAIS, and implements the risk assessment model through the Neural Network (NN) tool in MATLAB. Innovatively, a novel research perspective has been put forward; with the continuous development of Internet technology, Internet-based SCF is also rising; however, the relevant research in this field is far from being applied, and the research results are scattered; on the other hand, China has more research on traditional SC, there is a lack of research on the Credit Risk Evaluation (CRE) of Internet-based SCF; therefore, this paper tests the CRE model from the perspective of Internet-based SCF. Specifically, three research methods are applied: Backpropagation (BP) NN, Support Vector Machines (SVM), and Genetic Algorithm (GA). The research findings provide a certain reference for the development of SMEs.

## Construction of Internet-based SCF-oriented RAIS

The basic link of enterprise risk assessment is to build a reasonable credit RAIS. At present, the Internet is omnipresent. The emergence of SCF has helped SMEs alleviate their financial difficulties. The links between the Internet and the SC are becoming ever-closer [11, 12]. According to reasonable principles, indexes can be selected and used to build a complete and reasonable Internet-based SCF assessment system. The research idea is outlined in Fig 1:

**Fig 1:** The research ideas of this paper.

### Influencing factors of financial credit risk in Internet-based SC

The basic idea of CRE of Internet-based SCF is to provide financing services for SC. To evaluate the credit risk of SMEs in the SC, it is imperative to pay attention to the individual enterprise’s financial indexes but also the overall operation of the enterprise’s SC and the degree of information sharing. Additionally, it is necessary to use big data technology to obtain real-time transaction data and then make a systematic and scientific assessment of enterprise credit risk in the SC. This paper mainly analyzes the basic situation of the industry of SMEs that need financing and their own situation.

### SC financial risk assessment index

The enterprise Operational Excellence Index (OEI) can be divided into Debt-Paying Ability (DPA), Operation Ability (OA), and Profitability (P). DPA is generally described by Asset Liability Ratio (ALR), Current Ratio (CR), Interest Coverage Multiple (ICM), and Cash Asset Ratio (CAR), in which the ALR represents the ratio of an enterprise’s assets to liabilities; CR denotes the relationship between current assets and current liabilities of an enterprise; TIE is the ratio of the pretax profit of the enterprise to the loan interest of the enterprise [13, 14]; CR reflects the liquidity of the company’s assets. SMEs often pledge enterprise assets for bank credit lines to obtain loans; when they fail to pay on time (default), it will have an adverse impact on the bank. Therefore, this paper uses the amount and age of accounts receivable of financing enterprises to study the asset status of enterprises. The smaller the financial accounts receivable is, the lower the risk of accounting default is, and vice versa. With the continuous progress of Internet technology, more and more SC users can easily obtain the order data of financing enterprises in the SC. These data can be used to facilitate the analysis of the transaction behavior of enterprises [15, 16] and comprehensively monitor the enterprise risks. This practice can greatly improve the financing efficiency of enterprises and meet their financing needs. Thereupon, this paper selects the information level construction of the SC to analyze the development degree of the integration of Internet and SCF. The principle of this index is based on the development of enterprise SC searched on the Internet. The searched keywords are "name of SMEs" + "SC". According to the important role of index scale in the Analytical Hierarchy Process (AHP) scale system, this paper puts forward a four-level score assessment of 10/7/4/0 and uses four principles to select Internet-based SCF credit assessment indexes. They are the principles of objectivity and comprehensiveness: specifically, to make a more accurate credit assessment, there is a need to deeply consider the enterprise characteristics under the Internet-based SCF and the impact of the Internet on the SCF; the principle of operability, that is, the actual acquisition of data needs to be considered during index selection. Index data should be easy to collect and measure, and qualitative indexes should not add too many objective factors [17, 18]; the principle of independence is to avoid duplication of the information contained in indexes during index selection; the pertinence principle: during index selection, it is necessary to fully consider the business and mode of SCF stocks and select indexes that can comprehensively reflect the credit level of enterprises. According to these principles, the sub assessment indexes of the credit risk of SMEs selected, as shown in Table 1:

**Table 1:** Credit RAIS.

	1	2	3	Index description
A1	IS	IG	IGR/NPGR	Current/year-ago period
A2	MR	DPA	ALR	Assets/Liabilities
A3			CR	Current assets/current liabilities
A4			ICM	Profit before tax/interest expense
A5			CAR	(Cash + securities)/ current liabilities
A6		OA	IT	Cost of sales/average net inventory
A7			ART	Average balance of sales revenue/accounts receivable
A8			TAT	Sales revenue/average balance of assets
A9		P	NPOS	Net profit/operating income
A10			NPMOTA	Net profit/average balance of total assets
A11			ROE	Average balance of net profit/Stockholders’ equity
A12			GROTA	Current/previous year same period
A13	SIR	ARC	CARA	Proportion of accounts receivable less than one year
A14		ASOAR	DOIC	The degree to which transactions are realized online

In Table 1, Industry Status: IS; Industry Growth: IG; Income Growth Rate: IGR; Net Profit Growth Rate: HPGR; Subject Rating MR; Inventory Turnover: IT; Accounts Receivable Turnover: ART; Total Asset Turnover: TAT; Net Sales On Profit: NPOS; Net Profit Margin On Total Assets: NPMOTA; Return on Net Assets: ROE; Gross Asset Growth Rate: GROTA; Cautious Rating: SIR; Accounts Receivable Characteristics: ARC; Amount of Accounts Receivable in the Current Year: CARA; Aging Structure of Accounts Receivable: ASOAR; Degree of Information Construction: DOIC.

RETRACTED

According to the relevant research, if the correlation between the two indexes surpasses 0.6, they have a high correlation. The paper conducts correlation analysis on the selected 14 indexes, of which the correlation e between the growth rate of NPMOTA and NPOS is 0.76, and the ICM and CAR have a high correlation of 0.843. Therefore, after the correlation analysis of 14 preselected indexes, the two indexes of NPMOTA and ICM, the number of indexes of the Internet-based SCF CRE system is 12.

## SCF-oriented risk assessment method

### Analysis and implementation of Backpropagation Neural Network (BPNN) model

BPNN is a multi-layer forward network structure including the input layer, hidden layer, and output layer. The input layer receives signals; the hidden layer is responsible for the implicit transformation of signals; the output layer outputs the prediction results [19, 20]. The structure of BPNN is depicted in Fig 2.

**Fig 2:** BPNN structure.

The training process of BPNN can be divided into seven steps:

1. Network initialization is to determine the network parameters according to the network input sequence, such as the number of the input, hidden, and output layer nodes *n*, *l*, and *m*, as well as initialize the link weight *ω*_*i*,*j*_ and *ω*_*j*.*k*_ between neurons in each network layer, and finally, give the Learning Rate (LR) and Activation Function (AF).
2. Calculation of hidden layer output *H*_*i*_.
$$H_{i}=f\left(\overset{n}{\underset{i=1}{\sum }}\omega_{ij}x_{i}-a_{j}\right)j=1,2,\ldots ,l$$ (1)
  In Eq (1), *i* denotes the number of hidden nodes, *f* represents the excitation function of the hidden layer, *a* stands for the threshold of the hidden layer, and *ω*_*ij*_*x*_*i*_ means the link weight of the neural unit.
3. Output layer calculation is to calculate the prediction output *O*_*K*_ of BPNN.
$$O_{K}=\overset{l}{\underset{j=1}{\sum }}H_{j\omega_{jk}}-b_{k}$$ (2)
4. Error calculation is to calculate the prediction error *e* of the network.
$$e_{k}=Y_{k}-O_{K}$$ (3)
5. The link weights of neurons in the network are updated according to the network prediction error *b*.
$$\omega_{ij}=\omega_{ij}+\eta H_{j}\left(1-H_{j}\right)x\left(i\right)\overset{m}{\underset{k=1}{\sum }}\omega_{jk}e_{k}$$ (4)
$$\omega_{jk}=\omega_{jk}+\eta H_{j}e_{k}$$ (5)
6. Threshold update is to update the node threshold *a* and *b* according to the network prediction error *e*.
$$a_{j}=a_{j}+\eta H_{j}\left(1-H_{j}\right)\overset{m}{\underset{k=1}{\sum }}\omega_{jk}e_{k}$$ (6)
$$b=b_{k}+e_{k}$$ (7)
7. Judge whether the algorithm iteration ends; if not, return 2).

RETRACTED

### Analysis and implementation of Genetic Algorithm (GA) model

GA is a metaheuristic natural selection process, which belongs to evolutionary algorithms. It usually uses biological heuristics, such as mutation, crossover, and selection, to generate better optimization and search problem solutions. GA encodes the feasible solution of the problem into chromosomes to form an initial population and generates a new population through selection, crossover, mutation, and other operations. Only the fittest individuals in the new generation are retained to produce offspring of the next generation. Each new generation saves the information in the previous generation and outperforms its predecessors [21–23].

1. Encoding: GA is used to encode variables when solving problems. The expression for binary number conversion into decimal decoding reads:
$$F\left(b_{i1},b_{i2},b_{il}\right)=R_{i}+\frac{T_{i}-R_{i}}{2^{l}-1}\overset{l}{\underset{j=1}{\sum }}b_{ij}2^{j-1}$$ (8)
  In Eq (8), (*b*_*i1*_, *b*_*i2*_, …*b*_*il*_) is the i-th segment of each individual with a segment length of *1*, *T*_*i*_ and *R*_*i*_ mean the left and right endpoints of the definition domain of the *i*-th segment component, respectively; *j* stands for a natural number.
2. The fitness function can measure the fitness of individuals in the population.
3. The genetic operation can apply specific operations to individuals according to individual fitness to select the fittest individual. From the perspective of optimization search, the mutation operator improves the ability of GA to find the optimal solution [24–26]. The basic flow of GA is drawn in Fig 3:

**Fig 3:** Flowchart of GA.

### SVM model analysis and implementation

SVM is a supervised learning method for finite sample prediction and is proposed in the 1960s against the explicit linear separable problem. Generally, SVM cannot directly solve the high-dimensional problem, and the low-dimensional classification problem is transformed into high-dimensional space by introducing kernel function. Both linear regression and nonlinear regression belong to SVM regression [27, 28]. For linear regression, there is a function shown in Eq (9):

f(x)=ω⋅x+b (9)

The minimum value *ω* needs to be found to ensure the smoothness of Eq (9). Therefore, this paper assumes that there is a function *f* that can estimate all (*x*_*i*_, *y*_*i*_) within the accuracy *ε*, and solving the minimum value *ω* becomes a convex optimization problem, as shown in Eqs (10) and (11):

$${\text{min}}_{\omega ,b,\xi ,\xi^{*}}\frac{1}{2}\omega^{T}\omega +c\sum_{i=1}^{n}\left(\xi +\xi^{*}\right)$$ (10)

$$\xi^{*}=\{\begin{array}{l} 0,f\left(x_{i}\right)-y_{i}\leq \varepsilon \\ \left|f\left(x_{i}\right)-y_{i}\right|-\varepsilon ,\left|f\left(x_{i}\right)-y_{i}\right|\geq \varepsilon \end{array}$$ (11)

In Eq (10), *c* is the penalty factor.

RETRACTED

In solving the optimization problem, *c* is a fixed penalty factor; *c* represents the penalty strength of the model for the data beyond the interval *ε*. Eq (10) is transformed into a quadratic programming problem by using the duality principle, and the Lagrange equation is established, as shown in Eq (12):

$$l\left(\omega ,\xi_{i},\xi_{i}^{*}\right)=\frac{1}{2}{\left\|\omega \right\|}^{2}+C\left(\sum_{i=1}^{m}\xi_{i}+\xi_{i}^{*}\right)-\sum_{i}^{\infty }\alpha_{i}\left(\varepsilon +\xi_{i}-y_{i}+\left(\omega \cdot x_{i}\right)+b\right)-\sum_{i}^{\infty }\alpha_{i}^{*}\left(\varepsilon +\xi_{i}-y_{i}-\left(\omega \cdot x_{i}\right)-b\right)-\sum_{i=1}^{m}\eta_{i}\xi_{i}+\eta_{i}^{*}\xi_{i}^{*}$$ (12)

In Eq (12), the partial derivative of the parameter *ω*, *b*, *ξ*_*i*_, $\xi_{i}^{*}$ shall be equal to 0, which can be written as Eq (13):

$$\{\begin{array}{l} \frac{\partial l}{\partial \omega }=\omega -\sum_{i=1}^{m}\left(\alpha_{i}-\alpha_{i}^{*}\right)x_{i}=0\\ \frac{\partial l}{\partial b}=\sum_{i=1}^{m}\left(\alpha_{i}-\alpha_{i}^{*}\right)=0\\ \frac{\partial l}{\partial \xi_{i}}=C-\alpha_{i}-\eta_{i}=0\\ \frac{\partial l}{\partial \xi_{i}^{*}}=C-\alpha_{i}^{*}-\eta_{i}^{*}=0 \end{array}$$ (13)

The dual optimization problem is obtained by simplifying Eq (13), as shown in Eqs (14) and (15):

$$\text{min}\frac{1}{2}\sum_{i,j=1}^{m}\left(\alpha_{i}-\alpha_{i}^{*}\right)\left(\alpha_{j}-\alpha_{j}^{*}\right)\langle x_{i},x_{j}\rangle +\sum_{i=1}^{m}\alpha_{i}\left(\varepsilon -y_{i}\right)+\sum_{i=1}^{m}\alpha_{i}^{*}\left(\varepsilon +y_{i}\right)$$ (14)

$$\text{s}.\text{t}.\{\begin{array}{l} \sum_{i=1}^{m}\left(\alpha_{i}-\alpha_{i}^{*}\right)\\ \alpha_{i},\alpha_{i}^{*}\in [0,C] \end{array}$$ (15)

The relationship *ω* can be obtained by solving the shown in Eqs (14) and (15), as shown in Eq (16):

$$\omega =\sum_{i=1}^{N}\left(a_{i}+a_{i}^{*}\right)x_{i}$$ (16)

According to Karush-Kuhn-Tucker (KKT) theorem, there is the relationship shown in Eqs (17) and (18) at the optimal position.


$$\{\begin{array}{l} a_{i}\left(\varepsilon +\xi_{i}-y_{i}+\omega x+b\right)=0\\ a_{i}^{*}\left(\varepsilon +\xi_{i}^{*}-y_{i}+\omega x+b\right)=0 \end{array}$$ (17)

$$\{\begin{array}{l} \xi_{i}\left(C-a_{i}\right)=0\\ \xi_{i}\left(C-a_{i}^{*}\right)=0 \end{array}$$ (18)

Further, the relationship shown in Eq (19) can be obtained:

$$\omega =\sum_{i=1}^{m}\left(\alpha_{i}-\alpha_{i}^{*}\right)x_{i}$$ (19)

*f*(*x*) can be written as the relationship shown in Eq (20):

$$f(x)=\sum \left(\alpha_{i}-\alpha_{i}^{*}\right)\langle x_{i}\cdot x\rangle +b$$ (20)

In general, linear regression is solved under ideal conditions, but in actual prediction, there are many influencing factors, so it is necessary to introduce kernel function to map samples to high-dimensional space [29, 30]. Then, the optimization problem becomes the form shown in Eqs (21) and (22).


$$\omega \left(a,a^{*}\right)=-\frac{1}{2}\sum_{i,j=1}^{N}\left(a_{i}-a_{i}^{*}\right)\left(a_{j}-a_{j}^{*}\right)K\left(x_{i},x_{j}\right)+\sum_{i=1}^{N}\left(a_{i}-a_{i}^{*}\right)y_{i}-\sum_{i=1}^{N}\left(a_{i}+a_{i}^{*}\right)\varepsilon$$ (21)

$$\text{s}.\text{t}.\{\begin{array}{l} \sum_{i=1}^{N}\left(a_{i}^{*}-a_{i}\right)=0\\ 0\leq a_{i},a_{i}^{*}\leq \frac{C}{N},i=1,2,\ldots ,N \end{array}$$ (22)

By solving Eqs (21) and (22), the relationship as in Eqs (23) and (24) can be obtained:

$$\omega =\sum_{i=1}^{N}\left(a_{i}^{*}-a_{i}\right)\phi \left(x_{i}\right)$$ (23)

$$b=y_{i}-\sum_{i=1}^{N}\left(a_{i}^{*}-a_{i}\right)K\left(x_{i},x_{j}\right)-\varepsilon$$ (24)

The regression function is obtained as shown in Eqs (25) and (26):

$$f(x)=\sum_{i=1}^{N}\left(a_{i}-a_{i}^{*}\right)\left(\phi \left(x_{i}\right)\cdot \phi (x)\right)+b$$ (25)

$$f(x)=\sum_{i=1}^{N}\left(a_{i}-a_{i}^{*}\right)k\left(x_{i}\cdot x\right)+b$$ (26)

The nonlinear regression structure of SVM is shown in Fig 4:

**Fig 4:** SVM nonlinear regression.

RETRACTED

### Sample source and data analysis

ST is often used by scholars and relevant researchers to mark enterprises with such financial difficulties as debt default, while those enterprises without ST marks are recognized as healthy enterprises. This section chooses 16 enterprises with ST Mark and 84 enterprises with normal finance from 100 listed companies on China’s A-share SMEs board as modeling samples. All the sample quantitative data are from the Wind database [31, 32]. The data are transformed by Eq (27) to eliminate the need for standardization:

$$X_{i}^{\prime }=\frac{x_{i}-\text{min}(x)}{\text{max}(x)-\text{min}(x)}$$ (27)

In Eq (27), *x*_*i*_ is an individual of the sample *x*; max(*x*) stands for the maximum value in the sample *X*; min(*x*) indicates the minimum value in the sample, and $x_{i}^{\prime }$ means the transformed sample individual.

This paper involves three aspects of enterprise risks: high risk, medium risk, and low risk. The original data of SCF-oriented RAIS are shown in Table 2

**Table 2:** Original data of SCF-oriented RAIS.

Serial number	*A*_1_	*A*_2_	*A*_3_	*A*_4_	*A*_5_	*A*_6_	*A*_7_	*A*_8_	*A*_9_	*A*_10_	*A*_11_	*A*_12_	*A*_13_	*A*_14_
1	13.8	4	4	2	3	0.068	0.772	1.624	0.0305	0.726	50	3	3	3
2	13.8	3	3	3	4	0.061	4.032	1.352	0.152	2.514	32	2	2	4
3	13.8	4	4	4	4	0.087	5.912	1.891	0.014	1.150	30	3	3	3
4	13.8	3	4	4	3	0.085	2.119	1.24	0.071	3.854	90	3	3	2
5	13.8	4	2	1	4	0.3692	2.301	1.84	0.146	0.868	92	3	2	1

According to the above experimental data, this section uses the NN toolkit in MATLAB2016b to build a model with a parameter of 22 * 8 * 1 and eight hidden layer nodes. The AF of the hidden layer is Tansig [33], the AF of the output layer is Traingdx, the training times are 2,000, the LR is 0.01, and the target error is 0.001.

RETRACTED

The SVM algorithm and BPNN algorithm use the same data preprocessing methods to optimize the model performance. Here, 3,000 samples are used to build the SVM model; 2,000 samples are used to test the model; the Radial Basis Function (RBF) is selected as the kernel function of the SVM model.

The sample-set distribution is shown in Fig 5:

**Fig 5:** Sample set distribution.

## Algorithm test and simulation

### Results of SCF risk assessment

Table 3 shows the assessment results of the SCF-oriented RAIS based on the BPNN model.

**Table 3:** Test sample results.

	Model simulation results	Actual assignment
Risk assignment	0.362	0.333
Risk type	Low risk	Low risk

Table 3 illustrates that the risk assignment of the model simulation result is 0.362, the risk is low, and the actual assignment result is 0.333, the risk is low. Therefore, the assessment results of the proposed SCF-oriented RAIS mode based on BPNN are consistent with the actual sample, and the model has good risk assessment ability.

### Model classification and prediction results

The classification results of the SVM model (on a specific training process) are shown in Fig 6.

**Fig 6:** SVM model classification results (on a specific training process). ((a) SVM classification results on training set samples (b) SVM classification results on test set samples).

In Fig 6, *C*1*T* is the first test result of the actual classification of training set data, *P*1*T* represents the first test result of SVM model for the classification of training set data, *C*1*M* denotes the first test result of the actual classification of test set data, and *P*1*M* indicates the first test result of SVM model for the actual classification of test set data; *C*2*T* stands for the second test result of the actual classification of training set data, *P*2*T* means the second test result of the SVM model for the classification of training set data, *C*2*M* is the second test result of the actual classification of test set data, and *P*2*M* represents the second test result of SVM model for the actual classification of test set data; *C*3*T* is the third test result of the actual classification of training set data, *P*3*M* signifies the third test result of the SVM model on the classification of training set data, *C*3*M* refers to the third test result of the actual classification on test set data, and *P3M* stans for the third test result of SVM model for the actual classification on test set data. Apparently, after being trained by the training set, the classification effect of the SVM model on data is completely consistent with the actual classification effect. It can be proved that the learned SVM model is more suitable for the CRE of Internet-based SCF. In this experiment, the higher the coincidence degree between the classification curve of the actual test set is, and the classification curve of the predicted classification set is, the better the effect of the SVM model is. Fig 6(b) suggests that the data of only one sample point of the SVM model do not coincide, and the overall effect is excellent.

RETRACTED

This section randomly selects 100 different training sample sets and test sample sets for classification, and the output of classification results can be obtained, as shown in Fig 7:

**Fig 7:** SVM model experimental results (100 training samples). ((a) Partial classification results of SVM model training sample set (b) Partial classification results of SVM model test sample set).

As demonstrated in Fig 7(a), among all the classification results randomly selected here, the prediction results are completely consistent with the classification results from the historical data, and the classification accuracy of the training sample set is 97.2%. As indicated in Fig 7(b), for the random sampling prediction results, some prediction results are inconsistent with the actual situation, but the overall accuracy of the model prediction is high, which shows that the proposed RAIS and model are effective. The proposed model is tested multiple times. After 10 tests, the classification accuracy of the model to the training samples is 97.2%, and the classification accuracy of the model to the test samples is 96.2%.

Fig 8(a) and 8(b) show the actual classification and predicted classification results on the training sample set and the test sample set of the BP-GA model in a training process, respectively.

**Fig 8:** Experimental results of BP-GA model (on a training process). ((a) BP-GA model training sample set to predict classification results (b) Classification results of BP-GA model test sample set).

RETRACTED

The meaning of the legends in Fig 8 is similar to that in Fig 6, but the model is the BP-GA model.

Comparatively analysis of Figs 6(a), 6(b), 8(a) and 8(b) corroborates that the coincidence degree of classification results of the BP-GA model is better than that of the SVM model on the training data set; thus, BP-GA model is more suitable for the proposed Internet-based SCF-oriented RAIS.

Fig 9(a) depicts the classification results of the BP-GA model training sample set, and Fig 9(b) outlines the classification results of the BP-GA model test sample set.

**Fig 9:** Classification results of BP-GA model (100 training samples). ((a) classification results of BP-GA model on training sample set, (b) represents classification results of BP-GA model on test sample set).

Fig 9(a) implies that the predicted classification of the trained BP-GA model is completely consistent with the actual classification; the learned BP-GA NN model can be applied to the CRE of SCF. Fig 9(b) suggests that not all samples can be predicted accurately, but the performance of the model is still ideal.

### Algorithm comparison

The comparison of classification experiment results of SVM, BP model, and BP-GA model is shown in Fig 10:

**Fig 10:** Classification experimental results of SVM, BP model, and BP-GA model.

In Fig 10, 1 means the overall accuracy of the sample, 2 refers to the Type I error, and 3 indicates the Type II error. According to relevant research, when the model classifies an enterprise labeled as a defaulting enterprise as a performing enterprise, this kind of error is defined as the Type I error; by contrast, the Type II error is determined when the model classifies a performing enterprise into a defaulting enterprise. Compared with Type II error, Type I error causes greater losses to banks. Therefore, to investigate the performance of a classification model, there is a need to look at its overall classification accuracy but also to pay special attention to its Type I error rate. According to the comparison of classification results, the classification accuracy on test samples of BP, SVM, and BP-GA models are 82.33%, 95.31%, and 97.19%, respectively. The Type I error rates of the BP, SVM, and BP-GA models are 66.61%, 8%, and 7.2%, respectively. The Type II error rates of the BP, SVM, and BP-GA models are 7.4%, 14.29%, and 14.21%, respectively. Therefore, from the perspective of overall assessment accuracy, the BP-GA model is better than the BP model and SVM model.

## Conclusions

The core idea of SCF is to utilize the SC-dominating enterprises and their overall operation to increase credit for SC-affiliated enterprises. The identification and control of credit risk is the main link for banks to extend credit to SMEs. Therefore, it is imperative to discuss the relevant research details. With the maturity of SCF business, the expansion of enterprise participation scale, and the improvement of the enterprise information database, the SCF-oriented CRE will be easier to operate and more feasible. Therefore, there is a need to further adjust and improve the research details. Consequently, this paper puts forward the RAIS for SCF, establishes the SCF-oriented CRE system based on the GA-BP NN method, and verifies its effectiveness. The proposed model provides a standard for banks to judge the credit risk of upstream and downstream enterprises in the SC and speeds up the financing and borrowing speed of enterprises with good credit. Still, the proposed method has some shortcomings. Specifically, 1. The number of empirical samples is still insufficient. Mainly, enterprise credit data feature complex distribution, high dimensions, and relatively few samples. Although SVM can solve the problem of small samples, GA-BP model needs a large sample size. Too few samples will lead to biased parameter estimation and affect the model’s effectiveness. 2. Small sample volume will lead to seriously unbalanced sample distribution because the performing enterprises are easier to sample than the defaulting enterprises. Hence, if the sample category with a large number is eliminated, it will cause a waste of information and a shortage of training samples. 3. Sample collection is only limited to enterprises in Xi’an and the automobile industry SC, there is no corresponding research on the financial CRE of multi-regional and multi-industry SC. Moreover, the time span of the sample data is too short, so that the three indexes of legal and policy environment, industry development stage, and industry competition intensity cannot be included in the empirical research.

RETRACTED

## Supporting information

S1 Data (RAR)
